RETRACTED

# Clinical Features and Laboratory Examination Results of Sjogren's Syndrome Complicated with Thyroid Disorders: A Retrospective Analysis

**DOI:** 10.1155/2021/2280070

**Published:** 2021-10-29

**Authors:** Min Dai, Jing Wang, Qian Huang

**Affiliations:** ^1^Chongqing Hospital of Traditional Chinese Medicine, Chongqing 400021, China; ^2^Chongqing City Management College, Chongqing 401331, China

## Abstract

**Objective:**

To analyze the clinical incidence, clinical manifestations, laboratory examination, and complications of Sjogren's syndrome complicated with thyroid disorders in patients and to explore the clinical significance of its occurrence and concurrence relationship.

**Methods:**

The clinical manifestations, thyroid function, antithyroid antibodies, immunology indicators, autoantibodies, and routine laboratory examination items of 201 patients with Sjogren's syndrome in Chongqing Hospital of Traditional Chinese Medicine were reviewed and analyzed. According to whether the thyroid function was abnormal or not, the patients were divided into the group of Sjogren's syndrome complicated with abnormal thyroid function (*n* = 36) and the group of Sjogren's syndrome without abnormal thyroid function (*n* = 165). The clinical symptoms and test indicators of the two groups were compared.

**Results:**

Among 201 patients with Sjogren's syndrome, 36 patients had abnormal thyroid function (17.9%) and 36 patients with abnormal thyroid function had hypothyroidism. The abnormal renal function, decreased Hb, decreased WBC, increased ESR, and decreased C4 were more significant in the group with Sjogren's syndrome complicated with abnormal thyroid function, which had significant differences compared with the group with normal thyroid function (*P* < 0.05). The positive rates of aTG and aTPO in patients with Sjogren's syndrome complicated with thyroid disorders were higher than that in the normal group, and the difference between the two groups was statistically significant (*P* < 0.05).

**Conclusion:**

Patients with Sjogren's syndrome are often associated with hypothyroidism, and these patients may have more severe immune disorders, anemia, leukopenia, and renal involvement. The results show that paying attention to the detection of thyroid function in patients with Sjogren's syndrome may be of positive significance to judge the condition and prognosis.

## 1. Introduction

Sjogren's syndrome is a systemic chronic autoimmune disease mainly affected by exocrine glands such as the tear glands and salivary glands. Patients mostly show typical symptoms such as dry mouth and dry eyes. Sjogren's syndrome can be divided into primary and secondary categories according to the causes. Primary Sjogren's syndrome refers to connective tissue disease diagnosed without another diagnosis, and secondary Sjogren's syndrome refers to the disease associated with another clearly diagnosed connective tissue disease (such as systemic lupus erythematosus and rheumatoid arthritis). In abnormal thyroid disorders, autoimmune thyroid disease is a common organ-specific autoimmune disease, including Graves' disease, autoimmune thyroiditis/Hashimoto's disease, and primary hypothyroidism. The thyroid gland, salivary gland, and lacrimal gland are vulnerable to immune injury. For example, thyroiditis is a specific autoimmune disease involving a single organ. However, Sjogren's syndrome is a systemic autoimmune disease involving the salivary gland and lacrimal gland, and the two often coexist in clinical practice. Since adenoepithelial cells are the central target cells involved in autoimmune processes, Sjogren's syndrome is also known as “autoimmune epidermatitis” [1]. Sjogren's syndrome can affect multiple organs in addition to the involvement of exocrine glands, among which thyroid involvement is more common. More and more literatures suggest that [2] patients with Sjogren's syndrome have an expanding risk of autoimmune thyroid disease, and patients with autoimmune thyroid disease have an expanding risk of Sjogren's syndrome. Based on the analysis of the clinical data of Sjogren's syndrome patients hospitalized in the Rheumatology Department of Chongqing Hospital of Traditional Chinese Medicine, this paper discusses the clinical incidence, clinical manifestations, laboratory examination, and complications of Sjogren's syndrome complicated with thyroid dysfunction, focusing on the clinical characteristics and significance of Sjogren's syndrome complicated with thyroid dysfunction.

RETRACTED

## 2. Objects and Methods

### 2.1. Object of Study

A total of 201 patients diagnosed with Sjogren's syndrome admitted to the Department of Rheumatology, Chongqing Hospital of Traditional Chinese Medicine, from January 2013 to December 2017 were retrospectively analyzed. All patients were diagnosed following the International Classification of Sjogren's Syndrome (ICSJ) [3], revised in 2002. Among 201 patients with Sjogren's syndrome, there were 9 males (4.48%) and 192 females (95.52%), aged from 28 to 77 years, with an average of (54.40 ± 11.12) years. The course of the disease ranged from 3 months to 22 years. According to whether there was thyroid dysfunction, 201 patients with Sjogren's syndrome were divided into the group of Sjogren's syndrome with abnormal thyroid function (*n* = 36) and the group of Sjogren's syndrome without abnormal thyroid function (*n* = 165). The baseline levels of the two groups were homogeneous and comparable.

### 2.2. Clinical Data

The patient's basic information, clinical manifestations, complications, and laboratory tests were recorded. Basic information includes gender, age, and disease course. Clinical manifestations include dry mouth, dry eyes, arthralgia/arthritis, pulmonary interstitial lesions, and gastrointestinal symptoms. Complications: other rheumatoid diseases (rheumatoid arthritis, systemic lupus erythematosus, scleroderma, psoriasis, arthritis, ankylosing spondylitis, autoimmune liver disease, etc.). Laboratory tests include blood routine, liver and kidney function, erythrocyte sedimentation rate (ESR), c-reactive protein (CRP), immunoglobulin (IgG, IgM, and IgA), complement in blood serum (C3 and C4), thyroid function, thyroid antibody, and autoantibody spectrum. All the above indicators were routinely tested by the laboratory department of the hospital.

### 2.3. Statistical Method

SPSS26.0 statistical software was used for statistical analysis. If the measurement data conform to the normal distribution, it shall be expressed by mean ± standard deviation (*x* ± *s*). If the variance is homogeneous, two-independent sample *t*-test is used; if the variance is not homogeneous, two separate samples are tested as *T* prime test. If the data does not conform to the normal distribution, it is represented by the median (interquartile spacing) and two-independent sample rank-sum test is used. The counting data were expressed as cases and percentages, and the *χ*2 test was used for comparison. The *P* value less than 0.05 was used to indicate that the difference is statistically significant.

## 3. Results

### 3.1. Concurrent Disease and Thyroid Function of Patients

Among 201 patients with Sjogren's syndrome, 89 cases were complicated with other rheumatic immune diseases (77 cases of rheumatoid arthritis, 8 cases of systemic lupus erythematosus, 5 cases of scleroderma, 1 case of psoriatic arthritis, 1 case of ankylosing spondylitis, and 1 case of autoimmune liver disease) (Figure 1). According to the normal reference range of thyroid function index of TSH, respectively, 0.51–4.94 mIU/L, FT3 3.50–6.50 pmo l/L, FT4 12.25–21.78 pmo l/L, T4 58.1–140.6 pmo l/L; abnormal thyroid antibody reference for aTG >60 IU/ml and aTPO >60 IU/ml. Among 201 patients with Sjogren's syndrome, 36 cases (17.9%) had abnormal thyroid function, and 165 cases (81.9%) had normal thyroid function. 36 patients with abnormal thyroid function were classified as an abnormal group. We can find that all patients with abnormal thyroid function had hypothyroidism. The specific laboratory indexes for the diagnosis of hypothyroidism were abnormal FT3, FT4, and T4 with elevated TSH or only elevated TSH. No patients with hyperthyroidism were found.

RETRACTED

### 3.2. Clinical Manifestations

There was no significant difference in dry mouth, dry eyes, joint pain, pulmonary interstitial lesions, and gastrointestinal symptoms between 36 patients with Sjogren's syndrome complicated with abnormal thyroid function and 165 patients with normal thyroid function of Sjogren's syndrome (*P* > 0.05), as shown in Table 1.

### 3.3. Laboratory Inspection

There was no significant difference in liver function, immunoglobulin, platelet, CRP, and C3 between patients with Sjogren's syndrome combined with normal thyroid function and patients with Sjogren's syndrome combined with abnormal thyroid function (*P* > 0.05). The patients in Sjogren's syndrome combined with abnormal thyroid function group had more significant renal function abnormalities, decreased Hb, decreased WBC, increased ESR, and decreased C4, which were significantly different from those in the normal thyroid function group (*P* < 0.05), as shown in Table 2.

### 3.4. Autoantibody Level

There was no significant difference in the positive rates of antinatural SSA, antirecombinant SSA, and anti-SSB between the two groups (*P* > 0.05). Among 201 patients with Sjogren's syndrome, 74 cases of patients underwent aTG and aTPO. aTG positive patients were 14 (18.9%) and aTPO positive patients were 19 (25.6%). aTG and aTPO were detected in 24 patients with Sjogren's syndrome combined with abnormal thyroid function, of which 8 were ATG positive and 12 were aTPO positive. However, Among 50 patients with Sjogren's syndrome complicated with normal thyroid function, only 6 cases were ATG positive and 7 cases were aTPO positive. There was a significant difference in aTg and aTPO between the two groups (*P* < 0.05), as shown in Table 3.

## 4. Discussion

As we all know, autoimmune diseases have overlapping phenomena, that is, patients can suffer from one or more autoimmune diseases at the same time. In the study of the overlap of autoimmune diseases, it is found that among the patients with Sjogren's syndrome with abnormal thyroid function, the patients with Sjogren's syndrome and autoimmune thyroid diseases are the most common. At the same time, the most common cause of hypothyroidism is autoimmune thyroid disease, in which chronic lymphocytic thyroiditis, also known as Hashimoto's thyroiditis, is the most common, affecting about 10% of people in the world [4, 5]. Sjogren's syndrome is usually primary. However, many patients are often complicated with other autoimmune diseases, such as Hashimoto's thyroiditis, rheumatoid arthritis, and systemic lupus erythematosus [6], which is attributed to secondary Sjogren's syndrome. A recent review reported that the incidence rate of Sjogren's syndrome combined with autoimmune thyroid was 10–30% [7], which further showed that there were some connections and crossover between them. Sjogren's syndrome is less life-threatening, but it can cause severe symptoms such as dry mouth, dry eyes, and dental caries or affect the invasion of the lung, kidney, thyroid, and circulatory system, which will reduce the quality of life and even increase the risk of lymphoma. In this study, Sjogren's syndrome complicated with thyroid disorders in patients accounted for 17.9%. Hashimoto's thyroiditis is the most common autoimmune disease of Sjogren's syndrome [8]. Of course, it often coexists with other autoimmune diseases [9, 10]. In this study, there were 89 patients with Sjogren's syndrome complicated with other rheumatic immune diseases, including 20 cases in the abnormal thyroid function group and 69 cases in the normal group. There was no significant difference between the two groups, indicating that there was no significant relationship between Sjogren's syndrome complicated with abnormal thyroid function and other rheumatic immune diseases. It is suggested that thyroid function should be examined in both primary Sjogren's syndrome and secondary Sjogren's syndrome.

RETRACTED

Histologically and functionally, the thyroid gland, salivary gland, and lacrimal gland are very similar and are particularly vulnerable to immune injury. There is evidence that Sjogren's syndrome and autoimmune thyroid diseases have standard histopathological features [7]. Both diseases are characterized by focal or diffuse lymphocyte infiltration, especially CD4 T lymphocytes and activated B cells [9]. In autoimmune thyroid diseases, the role of epithelial cells in tissue inflammation and the presence of specific chemokines such as CXCL10 are considered to be markers of inflammatory response leading to tissue destruction. In particular, in Sjogren's syndrome, epithelial cells produce CXCL9 and CXCL10, resulting in salivary gland injury [7, 11].

In terms of genetic gene expression, Sjogren's syndrome and autoimmune thyroid diseases have the same linkage relationship with HLA-DR3/DR4 alleles. Some scholars found that the reaction of a certain region on the antihuman thyroglobulin antibody molecule in patients with Sjogren's syndrome and Hashimoto's thyroiditis overlapped, suggesting that this region is involved in the common pathogenesis of the two diseases [12].

Autoimmune thyroid diseases usually have aTG and aTPO levels rise. This study found aTG and the aTPO positive rates in Sjogren's syndrome. This study found that the positive rates of aTG and aTPO in patients with Sjogren's syndrome were 18.9% and 25.6%, respectively, which were basically similar to those reported in the literature. Patients with Sjogren's syndrome complicated with abnormal thyroid function are more likely to have positive thyroid antibodies than patients with Sjogren's syndrome complicated with normal thyroid function, which indicates that the leading cause of abnormal thyroid function in patients with Sjogren's syndrome is still the presence of thyroid antibody. The mechanism of this phenomenon is that thyroid antibodies combine with their own target antigens to form immune complexes, which deposit in the thyroid, and then activate lymphocytes to attack the thyroid so as to damage the thyroid function. Elevated thyroid antibody levels in patients with Sjogren's syndrome have been confirmed in some studies [9].

RETRACTED

The clinical characteristics of patients with Sjogren's syndrome complicated with autoimmune thyroid disease are unclear, and only a few cases have been reported [13, 14]. In our study, it was found that patients with Sjogren's syndrome complicated with abnormal thyroid function were more prone to anemia, decreased leukocyte, low C4, increased ESR, and abnormal renal function, suggesting that patients with Sjogren's syndrome complicated with autoimmune thyroid diseases may have more serious immune disorders. Studies have found that the level of serum IL-21 in patients with Sjogren's syndrome is increased, especially in patients complicated with hypothyroidism [15]. Through the cohort analysis of 723 patients with primary Sjogren's syndrome, it was found that low levels of C4 and purpura were the main risk factors for the development of primary Sjogren's syndrome into lymphoma [16].

Another study of 218 patients with primary Sjogren's syndrome also found that low C4 levels in these patients were associated with a high prevalence of peripheral neuropathy, cutaneous vasculitis, and lymphoma. At the same time, the study also reported that hypocomplementaemia, defined as low levels of C3, C4, or CH50, is also associated with higher mortality [17]. Whether this suggests that patients with Sjogren's syndrome complicated with abnormal thyroid function may have relatively high-risk factors for lymphoma remains to be further confirmed.

## 5. Conclusion

In conclusion, through the study of thyroid function in patients with Sjogren's syndrome and literature review, we preliminarily draw a conclusion: Sjogren's syndrome is often complicated with hypothyroidism and has a common physiological and pathological mechanism with autoimmune thyroid diseases. At the same time, such patients may have more serious immune disorders, more prone to anemia, leucopenia, and kidney involvement.

RETRACTED

Therefore, clinicians should make a comprehensive analysis in the diagnosis and treatment of Sjogren's syndrome to avoid missed diagnosis and misdiagnosis. In particular, when Sjogren's syndrome is complicated with anemia, leucopenia, and abnormal renal function, thyroid function should be checked routinely and treated in time. Similarly, clinicians should also be alert to autoimmune thyroid diseases and pay attention to the possibility of Sjogren's syndrome, so as to reduce missed diagnosis and misdiagnosis. However, our retrospective study has the disadvantages of a small sample size, many confounding factors, and missing data. At the same time, this study cannot determine the cause, but only the correlation. In the future research, more standard and standardized multicenter considerable sample investigation and analysis are needed to deeply reveal and confirm the clinical relationship of thyroid dysfunction in patients with Sjogren's syndrome.

## Figures and Tables

**Figure 1:** Complications in patients with Sjogren's syndrome.

**Table 1:** Clinical manifestations of the two groups.

Symptom	Normal group (165)	Abnormal group (36)	*X* ^2^	*P* value
Dry mouth	122	24	0.375	>0.05
Dry eye	98	17	0.181	>0.05
Joint pain	128	27	0.739	>0.05
Lung involvement	51	10	0.711	>0.05
Gastrointestinal tract involvement	54	13	0.696	>0.05

**Table 2:** Laboratory indexes of the two groups.

Project	Normal group (165)	Abnormal group (36)	*X* ^2^	*P* value
Liver function	22	4	0.719	>0.05
Renal function	14	11	0	<0.05
Hb	49	16	0.004	<0.05
PLT	21	5	0.851	>0.05
WBC	28	12	0.026	<0.05
CRP	34	9	0.56	>0.05
ESR	70	25	0.003	<0.05
IgG	54	10	0.748	>0.05
IgM	11	2	0.37	>0.05
IgA	26	11	0.062	>0.05
C3	36	13	0.07	>0.05
C4	4	4	0.016	<0.05

**Table 3:** Autoantibodies of the two groups.

Autoantibody	Normal group (165)	Abnormal group (36)	*X* ^2^	*P* value
Natural SSA	122	28	0.632	>0.05
Restructuring of SSA	99	26	0.171	>0.05
SSB	10	10	0.225	>0.05
aTG	6	8	0.028	<0.05
aTPO	7	12	0.001	<0.05
Overlap	69	20	0.143	>0.05

## Data Availability

The simulation experiment data used to support the findings of this study are available from the corresponding author upon request.
